RETRACTED

# Long non-coding RNA MALAT1 aggravated liver ischemia-reperfusion injury via targeting miR-150-5p/AZIN1

**DOI:** 10.1080/21655979.2022.2073124

**Published:** 2022-06-05

**Authors:** Qiang Sun, Jinlong Gong, Xueyi Gong, Jianlong Wu, Zhipeng Hu, Qiao Zhang, Xiaofeng Zhu

**Affiliations:** a General Surgery Department 1, Zhongshan People’s Hospital, Zhongshan Hospital of Sun Yat-sen University, Zhongshan, Guangdong, China; b Organ Transplant Center, The First Affiliated Hospital, Sun Yat-sen University, Guangzhou, Guangdong, China

**Keywords:** MALAT1, miR-150-5p, liver ischemia/reperfusion injury, AZIN1

## Abstract

Long non-coding RNA (lncRNA) metastasis-associated lung adenocarcinoma transcript 1 (MALAT1) plays a crucial role in the process of renal ischemia-reperfusion (IR) injury and myocardial IR injury. However, its mechanism in liver IR injury is not clear. IR and hypoxia/reoxygenation (H/R) model were built on C57BL/6 mice. Blood samples were obtained from the inferior vena cava of the model mice. MALAT1 expression was detected in IR model and H/R model. Supported by experimental results, the impacts of MALAT1 on viability, apoptosis, and inflammation of H/R model cells were detected. The correlation between MALAT1 and downstream genes was analyzed by mechanism assays. MALAT1 was detected to be upregulated in IR model and H/R model. MALAT1 knockdown had inhibitory effects on apoptosis and inflammatory reaction while promoting liver cell viability in H/R condition. Meanwhile, MALAT1 targeted miR-150-5p to regulate antizyme inhibitor 1 (AZIN1) in liver cells. Finally, MALAT1 regulated viability, apoptosis, and inflammatory reaction of liver cells by targeting miR-150-5p and AZIN1. To conclude, MALAT1 targeted miR-150-5p/AZIN1 to accelerate liver IR injury, suggesting that MALAT1 might be a novel target for liver IR injury.

## Highlights

- MALAT1 is up-regulated in liver IR injury models.
- MALAT1 affects viability, apoptosis and inflammatory response of H/R model.
- MALAT1 promotes liver IR injury via miR-150-5p/AZIN1 axis.

## Introduction

Ischemia-reperfusion (IR) is a common pathological process in various organs. It not only had little work on recovering the physical function of an organ but also damaged the structure [1]. Microcirculation disorder, excessive oxygen free radicals, and apoptosis are important mechanisms of hepatic injury [2]. During the period of reperfusion, dysfunctional tissue produces reactive oxygen species, which activates apoptosis mediators and inflammatory processes [3]. Liver IR injury is an inevitable complication occurring during liver surgeries [4]. Such injury is induced by a complex cascade of inflammatory mediators, which could recruit activated leukocytes into the liver [5]. Therefore, it requires intense commitment and efforts for in-depth exploration of IR injury.

RETRACTED

Long non-coding RNAs (lncRNAs) possessing a length of over 200 nucleotides have only limited protein-coding capacities [6], but this group of RNAs has been suggested as crucial effectors implicated in development and progression of diseases including cancers. For example, PANDAR has been suggested to predict poor prognosis and accelerate the progression of cervical cancer [7]. Erbb-IR accelerates diabetic kidney injury via sponging miR-29b [8]. MEG3 is identified as a valuable target in hepatic IR [9]. Likewise, metastasis-associated lung adenocarcinoma transcript 1 (MALAT1) has been suggested as a crucial participant in spinal cord IR injury and myocardial IR injury [10][11]. We established a liver IR model and discovered that MALAT1 expression was elevated after IR treatment. Therefore, it is worthwhile to explore the role of MALAT1 in liver IR injury.

Accumulating evidence indicates that lncRNAs can function as competitive endogenous RNAs (ceRNAs), and specifically, lncRNAs serve as miRNA sponge to lessen the bond between miRNAs and their downstream mRNAs, thereby leading to the release of protein-coding of mRNAs [12]. Recent researches have uncovered the lncRNA-miRNA-mRNA ceRNA networks implicated in the progression of multiple diseases [13]. In terms of IR injury, it has been found that CHRF affects the development of cerebral IR injury through miR-126/SOX6 axis [14]. Besides, HOTAIR acts as a ceRNA to modulate autophagy via sequestering miR-20b-5p to regulate ATG7 in hepatic IR injury [15]. In addition, lncRNA NORAD is proved to protect against IR injury-induced cell apoptosis, oxidative stress, brain damage, and inflammation via miR-30a-5p/YWHAG axis [16]. However, the potential ceRNA network of MALAT1 essential to liver IR injury remains to be elucidated.

Collectively, we mainly intended to unveil the implication of MALAT1 in liver IR injury. Thus, experiments with hypoxia/reoxygenation (H/R) model of liver immortalized cell lines and primary mouse hepatocytes were designed to identify the role and potential ceRNA mechanism of MALAT1. With all our efforts, we intended to provide a novel sight for understanding liver IR.

## Materials and methods

### Hepatic IR injury model

The hepatic IR injury model was strictly constructed [17]. The animal-related experiments were implemented with the approval of the Animal Research Committee of Zhongshan People’s Hospital, Zhongshan Hospital of Sun Yat-sen University. Male C57BL/6 mice (6–8 weeks old), obtained from Vital River Laboratory Animal Company (Beijing, China), were anesthetized by 50 mg/kg of pentobarbital sodium in order to construct the mice model of 70% partial hepatic ischemia. The middle and left hepatic pedicles of mice, including the portal vein, hepatic pedicles, and bile duct, were clamped for 1 h after midline laparotomy. After the remaining hepatic lobe blood vessel was retained, samples were examined for reperfusion after 2, 4, 6, and 10 h for experimental determination.

RETRACTED

### Primary hepatocyte isolation

Primary hepatocytes were isolated from IR model with a two-step perfusion method according to the procedures described in previous research [18]. Isolated hepatocytes were seeded on collagen-coated culture dishes and then obtained for conducting indicated experiments on the following day.

### Serum sample test

Blood samples obtained from the inferior vena cava of C57BL/6 mice were preserved for 20 min at 4°C, centrifuged for 10 min at 3000 × g at 4°C, and then, 4 ml of serum sample was extracted. The levels of liver enzymes and pro-inflammatory cytokines in serum samples were measured. Specifically, ELISA kits obtained from R&D Systems (Minneapolis, MN, USA) and Foreland Pharma Biological Technology (Beijing, China) were, respectively, used for detecting levels of tumor necrosis factor alpha (TNF-α) and interleukin-6 (IL-6) and for aspartate aminotransferase (AST) and alanine aminotransferase (ALT). The absorbance was measured at 450 nm with a microplate reader (Model 680; Bio-Rad, Hercules, CA, USA).

### Cell culture

Liver immortalized cell lines THLE-2 and THLE-3, available from ATCC (Manassas, VA, USA), were allowed to culture in the BEGM (Lonza/Clonetics Corporation, Walkersville, MD, USA). The 10% fetal bovine serum and 1% penicillin-streptomycin both procured from Gibco (Grand Island, NY, USA) were used to supplement cell culture medium. An environment with 5% CO_2_ at 37°C was maintained for culture of cells.

### H/R model

The construction of H/R model was strictly based on the steps described in previous literature [19]. Briefly, the culture dishes in chamber were subjected to treatment with AnaeroPack-Anaero (MGC, Tokyo, Japan) as the oxygen absorber-CO_2_ generator, following the established protocol. The oxygen indicator was utilized for assessment of the oxygen concentration, and it turned pink under the indicated condition: O_2_ concentration < 5%. After the chamber was placed in the cell culture incubator for 3 h, the reoxygenation was conducted via transferring the plates from hypoxic chamber to the normoxic, humidified incubator for 2, 4, 6, and 10 h. Both normoxic and hypoxic treatments were undertaken at 37°C.

### Reverse transcription quantitative real-time polymerase chain reaction (RT-qPCR)

RT-qPCR was done for measurement of indicated genes in accordance with the procedures described in previous literature [20]. Total RNA was initially isolated from tissues and cells with TRIzol Reagent (Invitrogen, Carlsbad CA, USA). Thereafter, PrimeScript Reverse Transcriptase Kit was used for cDNA synthesis, as guided by provider (Takara, Shiga, Japan). Gene expression was examined by SYBR Green PCR Kit (Takara) via RT-qPCR and calculated following the 2^−ΔΔCt^ method. Glyceraldehyde-3-phosphate dehydrogenase (GAPDH) or U6 was employed as the internal reference. Primer sequences used are listed in Supplementary file 1.

RETRACTED

### Cell transfection

The specific shRNAs to MALAT1 for knocking down MALAT1, as well as nonspecific shRNAs (negative control; NC), were provided by GenePharma (Shanghai, China). The full-length cDNA sequences of MALAT1 and AZIN1 were, respectively, inserted into the pcDNA3.1 vectors (Invitrogen) for overexpressing the indicated genes, and the empty vector (pcDNA3.1) was used as control. Additionally, miR-150-5p mimics and NC mimics were synthesized by Ribobio (Guangzhou, China). The abovementioned plasmids were, respectively, transfected or co-transfected into THLE-2, THLE-3, and primary mouse hepatocytes for 48 h with Lipofectamine 3000 (Invitrogen).

### Cell counting kit-8 (CCK-8) assay

CCK-8 assay was done with transfected liver immortalized cell lines and primary mouse hepatocytes, together with the CCK-8 assay kit (Dojindo Laboratories, Kumamoto, Japan) in accordance with procedures described in recent research [21]. Cells seeded in 96-well plates (5 × 10^3^ cells/well) were incubated with 10 μL of CCK-8 solution for 2 h. Then, the absorbance at 450 nm was examined with spectrophotometer (Thermo Fisher Scientific, Waltham, MA, USA).

### Flow cytometry

Flow cytometry assay was done with reference to a previous study [22]. 1 × 10^6^ cells (THLE-2, THLE-3, and primary mouse hepatocytes) were collected after transfection and then placed into 6-well plates. Flow cytometer (BD Biosciences, Franklin Lakes, NJ, USA) and the Annexin V-FITC/PI double staining kit (Invitrogen) were procured for the implementation of this assay. After 15-min staining, cell samples were reaped for flow cytometry. As the gating strategy used in flow cytometry analysis, FSC (forward scatter) and SSC (side scatter) thresholds were set to remove debris or noise. The raw data is included in Supplementary file 2.

### Terminal-deoxynucleotidyl transferase-mediated nick end labeling (TUNEL) assay

TUNEL assay was done with TUNEL reagent (Merck KGaA, Darmstadt, Germany) following procedures described in previous study [23]. The transfected cells (1 × 10^4^) including THLE-2, THLE-3, and primary mouse hepatocytes seeded in 96-well plates were subjected to fixation in 4% paraformaldehyde. After permeabilization with 0.1% Triton-X100, cells were treated with TUNEL kit, followed by nuclear staining with DAPI staining. Olympus fluorescence microscope (Tokyo, Japan) was used for observation.

RETRACTED

### Caspase-3 activity assay

Beyotime C1115 Caspase 3 Activity Assay Kit (Shanghai, China) was procured for detection of caspase-3 activity, and the procedures in previous study were followed [24]. Cell protein extracts were prepared to incubate with caspase-3 substrate and assay buffer for 4 h. Finally, the absorbance was determined at 405 nm by spectrophotometer (Thermo Fisher Scientific).

### Fluorescent in situ hybridization (FISH)

FISH assay was conducted with specific RNA probe (Ribobio) for determining the cellular distribution of MALAT1 in THLE-2 and THLE-3 as previously performed [25]. Cells fixed in 4% paraformaldehyde were collected and washed, followed by hybridization with MALAT1-probe. Hoechst solution was added for staining cell nuclei. The fluorescent images were acquired with fluorescence microscope.

### Nuclear cytoplasm fractionation

Cytoplasmic and Nuclear RNA Purification Kit (Norgen, Thorold, ON, Canada) was acquired for detecting cellular accumulation of MALAT1, and the procedures were in accordance with published literature [26]. The lysed cells in cell fractionation buffer were collected for centrifugation. MALAT1 content in cell cytoplasm and nucleus was separately detected by RT-qPCR, with GAPDH and U6 used as controls.

### RNA pull-down assay

RNA pull-down assay was done with Pierce Magnetic RNA-Protein Pull-Down Kit (Thermo Fisher Scientific) in accordance with procedures described in previous literature [27]. The cell protein lysates were mixed with biotinylated MALAT1 or AZIN1 containing the wild-type (WT) and mutant (Mut) binding sites of miR-150-5p, followed by the addition of 30 μl of magnetic beads for another 2-h incubation. RNA-protein mixture was analyzed using RT-qPCR.

### Luciferase reporter assay

Luciferase reporter assay was implemented following strict procedures [28]. The fragments of MALAT1 or AZIN1 covering WT and Mut miR-150-5p binding sites were acquired and cloned into pmirGLO dual-luciferase plasmid (Promega, Madison, WI, USA) for constructing MALAT1-WT/Mut and AZIN1-WT/Mut. Then, the constructs were co-transfected with indicated plasmids into THLE-2 and THLE-3 cells for 48 h. Dual-luciferase reporter assay system (Promega) was used for assessing the luciferase activity in cells under different transfection conditions. Renilla expression vector served as a normalized control.

RETRACTED

### RNA immunoprecipitation (RIP)

Magna RIP™ RNA-Binding Protein Immunoprecipitation Kit was available from Millipore (Bedford, MA, USA) for conducting RIP assay based on standard procedures [21]. The cell lysates collected from RIP lysis buffer were conjugated with human Ago2 antibody or control IgG antibody and magnetic beads. After that, the immunoprecipitates were analyzed via RT-qPCR.

### Statistical analyses

Data were displayed as the means ± standard deviation from three independently conducted assays. The statistical analysis in form of analysis of variance or Student’s t-test was achieved by use of GraphPad PRISM 6 (GraphPad, San Diego, CA, USA). P-value < 0.05 was taken to indicate the statistical significance.

## Results

We mainly intend to fathom out the functional role of MALAT1 in liver IR injury with utilization of a liver IR injury model and H/R model of liver immortalized cell lines THLE-2 and THLE-3. ALT, AST, TNF-α, and IL-6 levels were detected via ELISA to reflect IR injury level after reperfusion of different time periods. Expression of MALAT1 was determined in constructed models. Proliferation and apoptosis as well as the inflammation of cells with H/R treatment and different transfections were evaluated to analyze the functional roles of genes. It was hypothesized that cytoplasmic MALAT1 could affect liver IR injury via acting as a ceRNA. Mechanism assays were done to analyze the ceRNA axis.

### MALAT1 is upregulated in liver IR injury model

To probe into the implication of MALAT1 in liver IR injury, we constructed a liver IR model in mice. The detailed process of IR model was constructed as follows: hepatic ischemia for roughly 1 h and subsequently reperfusion for 2, 4, 6, and 10 h at room temperature. All mice were sacrificed after reperfusion. Their liver and serum were collected and analyzed. As exhibited in Figure 1(a-b), the levels of serum ALT and AST were detected to be the highest after 6-h reperfusion. Meanwhile, the concentration of inflammatory cytokine (IL-6 and TNF-α) was also detected to increase, especially after 6-h reperfusion in IR model (Figure 1c-d). These results suggested that liver IR model was most successfully built when the reperfusion lasted for 6 hours. We also detected the expression of MALAT1 in IR model with 6-h reperfusion and found MALAT1 level displayed a remarkable higher level in IR model compared with sham model (Figure 1(e)). In short, MALAT1 expression was upregulated in liver IR mouse model.

**Figure 1.** **MALAT1 is upregulated in liver IR injury model**. (a-b) Levels of ALT and AST in serum samples from IR injury model versus the sham group mice were measured. n = 3. (c-d) Inflammatory cytokines (IL-6 and TNF-α) in serum samples from mice livers after IR treatment compared with sham group were analyzed. (e) MALAT1 expression was detected in IR injury by RT-qPCR. *P < 0.05, **P < 0.01.

RETRACTED

### Downregulated MALAT1 regulates liver cell viability, apoptosis rate, and inflammatory responses after H/R treatment

Next, liver cells THLE-2 and THLE-3 were subjected to 3-h hypoxia (5% O_2_), followed by reoxygenation (21% O_2_) for 2, 4, 6, and 10 h) at room temperature. RT-qPCR data revealed that MALAT1 expression was enhanced after 4-h and 6-h reoxygenation, while no significant difference was observed upon 2-h or 10-h reoxygenation (Figure 2(a)). In addition, 6-h reoxygenation after 3-h hypoxia was determined to be the optimum treatment and chosen for subsequent experiments. Then, we used sh-MALAT1#1/2 to knock down MALAT1 in THLE-2 and THLE-3 cells, and RT-qPCR verified the efficiency of MALAT1 silencing (Figure 2(b)). Additionally, primary hepatocytes were isolated from IR mouse model with 6-h reperfusion, and sh-MALAT1#1/2 was also transfected into primary mouse hepatocytes to silence MALAT1. RT-qPCR indicated that the sh-MALAT1#1/2 could effectively deplete the expression of MALAT1 in primary mouse hepatocytes (Fig. S1A). Results of CCK-8 assay revealed that H/R-treated cell viability was increased due to downregulation of MALAT1 (Figure 2(c) & Fig. S1B). From flow cytometry and TUNEL assay results, cell apoptosis was found to be lessened by knockdown of MALAT1 (Figure 2(d-e) & Fig. S1C-D). Moreover, caspase 3 activity was decreased by MALAT1 downregulation (figure 2(f) & Fig. S1E), and IL-6 and TNF-α were diminished after downregulation of MALAT1 (Figure 2(g-h) & Fig. S1F-G). Altogether, MALAT1 inhibited the viability of liver cells with H/R treatment while promoting apoptosis and inflammatory response.

**Figure 2.** **Downregulated MALAT1 affects viability, apoptosis and inflammatory responses of H/R model**. THLE-2 and THLE-3 cells were subjected to reoxygenation for indicated periods (2, 4, 6, and 10 h) after 3-h hypoxia treatment. (a) RT-qPCR evaluated MALAT1 expression in THLE-2 and THLE-3 cells with indicated treatment. H/R model after 3-h hypoxia and 6-h reperfusion was chosen for subsequent experiments. (b) MALAT1 expression in sh-MALAT1#1/2-transfected THLE-2 and THLE-3 cells was detected via RT-qPCR. (c) THLE-2 and THLE-3 viability was tested by CCK-8 after transfection of sh-MALAT1#1/2. (d-e) Apoptosis of sh-MALAT1#1/2-transfected THLE-2 and THLE-3 was assessed by flow cytometry analysis and TUNEL assays. (f) Caspase 3 activity in THLE-2 and THLE-3 cells transfected with sh-MALAT1#1/2 was examined with caspase 3 activity assay kit. (g-h) Supernatants of THLE-2 and THLE-3 cells transfected with sh-MALAT1#1/2 were collected to measure TNF-α and IL-6 by ELISA. *P < 0.05, **P < 0.01, n.s. meant no significance.

RETRACTED

### MiR-150-5p binds to MALAT1 in liver cells

To further explore the regulatory mechanism regarding MALAT1, we conducted FISH and nuclear cytoplasm fractionation assay to determine the subcellular distribution of MALAT1, and the major cytoplasmic accumulation of MALAT1 was ascertained (Figure 3(a-b)). It implied that MALAT1 might function via post-transcriptional regulation in liver cells. CeRNA mechanism, considered as a common post-transcriptional modulatory network, plays an important role in cellular processes [29]. We guessed MALAT1 might act as a ceRNA in liver cells. To verify our assumption, we searched on starBase (http://starbase.sysu.edu.cn) database for miRNAs possible to bind with MALAT1, and 5 miRNAs were screened out as the candidates under indicated conditions (CLIP Data: strict stringency (≥5); Degradome Data: high stringency (≥3); Pan-Cancer: 4 cancer types). We measured candidate miRNA levels in THLE-2 and THLE-3 cells in control group or after 6-h reoxygenation. RT-qPCR data demonstrated that after reoxygenation, only miR-150-5p expression reduced compared with normal controls (Figure 3(c)). Therefore, we chose miR-150-5p as our research target. The binding sites of MALAT1 and miR-150-5p predicted on starBase database are shown in Figure 3(d). For further verifying the binding between MALAT1 and miR-150-5p, RNA pull-down assays were conducted, the results of which manifested that biotinylated MALAT1-WT, instead of biotinylated MALAT1-Mut, could substantially pulled down miR-150-5p (Figure 3(e)). Moreover, we overexpressed miR-150-5p in THLE-2 and THLE-3 cells by miR-150-5p mimics transfection (figure 3(f)). Luciferase reporter assay was conducted with cells after co-transfection of miR-150-5p mimics and MALAT1-WT/Mut, and it was observed that miR-150-5p augment could only contribute to inhibited luciferase activity of MALAT1-WT but had little influence on that of MALAT1-Mut (Figure 3(g)). In conclusion, miR-150-5p bound to MALAT1 in liver cells.

**Figure 3.** **MiR-150-5p binds to MALAT1 in liver cells**. (a-b) FISH and nuclear cytoplasm fractionation experiments were done for determining subcellular accumulation of MALAT1. (c) The expression levels of five candidate miRNAs potentially binding to MALAT1 were detected by RT-qPCR in H/R model (6 h reperfusion) and in the control group. (d) starBase predicted binding sites between MALAT1 and miR-150-5p. (e) RNA pull-down assay validated the combination between miR-150-5p and MALAT1. ‘UUGGGAG’ was MALAT1-WT and ‘AACCCUC’ was MALAT1-Mut. (f) MiR-150-5p expression was assessed in THLE-2 and THLE-3 cells transfected with miR-150-5p mimics. (g) Luciferase reporter assays were done to verify the validity of the predicted binding sites of MALAT1 and miR-150-5p. ‘UUGGGAG’ was MALAT1-WT and ‘AACCCUC’ was MALAT1-Mut. **P < 0.01, n.s. meant no significance.

RETRACTED

### MiR-150-5p regulates liver cell viability, apoptosis, and inflammatory reaction after H/R treatment

Afterward, the effects of miR-150-5p on liver cells under the condition of H/R were analyzed. First, miR-150-5p was found to be significantly downregulated at 6 h after reoxygenation, and 6-h reoxygenation was selected for constructing H/R model used in subsequent experiments (Figure 4(a)). Then, we performed functional assays to observe miR-150-5p influences on H/R-treated cells. CCK-8 assay unveiled that miR-150-5p upregulation enhanced cell viability (Figure 4(b)). Through flow cytometry and TUNEL assays, we discovered that cell apoptosis was lessened in response to miR-150-5p augment (Figure 4(c-d)). After detection of caspase 3 activity, we also found miR-150-5p overexpression could decrease caspase 3 activity (Figure 4(e)). Moreover, IL-6 and TNF-α levels were found to decline upon miR-150-5p upregulation (figure 4(f-g)). To sum up, miR-150-5p had promoting influence on proliferation and inhibitory influence on apoptosis and inflammatory reaction of liver cells after H/R treatment.

**Figure 4.** ***MiR-150-5p regulates viability, apoptosis and inflammatory reaction of H/R model.*** THLE-2 and THLE-3 cells treated with 3-h hypoxia were subjected to reoxygenation treatment for indicated periods (2, 4, 6, and 10 h). H/R model with 6-h reperfusion was selected. (a) MiR-150-5p expression was examined in H/R model. (b) Cell viability was examined in H/R model with transfection of miR-150-5p mimics. (c-d) Apoptosis rate of cells upon miR-150-5p mimics or NC mimics transfection was evaluated with flow cytometry analysis and TUNEL. (e) Caspase 3 activity was examined in cells upon miR-150-5p mimics or NC mimics transfection. (f-g) IL-6 and TNF-α levels upon miR-150-5p mimics or NC mimics transfection were assessed by ELISA. *P < 0.05, **P < 0.01, n.s. meant no significance.

### AZIN1 is targeted by miR-150-5p

We further explored the downstream of miR-150-5p. 4 mRNAs with potential to bind with miR-150-5p were predicted on starBase (CLIP Data: strict stringency (≥5); Degradome Data: high stringency (≥3); Pan-Cancer: 10 cancer types). After transfecting miR-150-5p mimics into THLE-2 and THLE-3 cells, we discovered that only AZIN1 expression was strikingly reduced, whereas the expression of other mRNAs had no obvious changes (Figure 5(a)). Then, binding sites of miR-150-5p and AZIN1 predicted on starBase are displayed in Figure 5(b). To verify the effectiveness of the binding sites, RNA pull-down assays were carried out. It was manifested that miR-150-5p could be substantially pulled down by Bio-AZIN1-WT instead of Bio-AZIN1-Mut (Figure 5(c)). The results evidenced that AZIN1 and miR-150-5p bound at the predicted sites. Furthermore, it was manifested in RIP data that AZIN1, miR-150-5p, and MALAT1 were substantially precipitated in Anti-Ago2, further indicating the existence of a ceRNA network involving MALAT1, miR-150-5p, and AZIN1 (Figure 5(d)). Luciferase reporter assay was conducted for confirmation. In preparation, pcDNA3.1/MALAT1 was transfected into THLE-2 and THLE-3 cells to overexpress MALAT1, and RT-qPCR certified the overexpression efficiency was high (Figure 5(e)). The result of luciferase reporter assay showed that the luciferase activity of AZIN1-WT weakened upon miR-150-5p overexpression was recovered after co-transfection of pcDNA3.1/MALAT1, while that of AZIN1-Mut group hardly varied, which further illustrated the competing relationship between AZIN1 and MALAT1 on the binding sites of miR-150-5p (figure 5(f)). In a word, AZIN1 was the downstream target of miR-150-5p.

RETRACTED

**Figure 5.** **AZIN1 is the downstream target of miR-150-5p**. (a) Four mRNAs expressions were detected in THLE-2 and THLE-3 cells after miR-150-5p mimics transfection. (b) Binding sites between AZIN1 and miR-150-5p were predicted on starBase website. (c) RNA pull-down assay detected the combination between AZIN1 and miR-150-5p. ‘UGGGAG’ was AZIN1-WT and “ACCCUC” was AZIN1-Mut. (d) In RIP assay, RT-qPCR was done for measuring the enrichment of AZIN1, miR-150-5p and MALAT1 in Anti-Ago2. (e) MALAT1 expression was evaluated by RT-qPCR in pcDNA3.1/MALAT1-transfected THLE-2 and THLE-3. (f) Luciferase reporter assays corroborated the competing relationship between AZIN1 and MALAT1 on miR-150-5p binding sites. **P < 0.01, n.s. meant no significance.

### AZIN1 upregulation offsets the impacts of MALAT1 downregulation on in vitro liver IR injury model

To investigate whether MALAT1 regulated AZIN1 to affect liver IR injury, we carried out rescue assays with H/R cell model. We used pcDNA3.1/AZIN1 to increase the expression of AZIN1, and RT-qPCR proved the overexpression efficiency was high (Figure 6(a)). Then, THLE-2 and THLE-3 cells with H/R treatment were transfected with sh-NC, sh-MALAT1#1, or sh-MALAT1#1+ pcDNA3.1/AZIN1, respectively. It was manifested in CCK-8 assay that cell viability strengthened by MALAT1 downregulation was fully countervailed by overexpression of AZIN1 (Figure 6(b)). Through flow cytometry analysis and TUNEL assay, it was discovered that cell apoptosis weakened by MALAT1 silence was completely recovered by co-transfection of pcDNA3.1/AZIN1 (Figure 6(c-d)). Moreover, upregulated AZIN1 totally offset the inhibitory impacts of MALAT1 depletion on the caspase 3 activities (Figure 6(e)). Additionally, decrease in IL-6 and TNF-α concentration resulting from MALAT1 knockdown was almost reversed by AZIN1 overexpression (figure 6(f-g)). To summarize, MALAT1 accelerated liver IR injury of in vitro model by enhancing AZIN1.

RETRACTED

**Figure 6.** **AZIN1 upregulation offsets the impacts of MALAT1 downregulation on IR injury**. THLE-2 and THLE-3 cells were subjected to 3-h hypoxia and then 6-h reoxygenation. (a) AZIN1 expression in pcDNA3.1/AZIN1-transfected THLE-2 and THLE-3 cells was tested by RT-qPCR. Rescue experiments were performed with THLE-2 and THLE-3 cells transfected with sh-NC, sh-MALAT1#1 and sh-MALAT1#1+ pcDNA3.1/AZIN1. (b) CCK-8 examined cell viability in these three groups. (c-d) Apoptosis of cells with indicated transfection was evaluated by flow cytometry and TUNEL assays. (e) Caspase 3 activity was assessed in these three groups. (f-g) IL-6 and TNF-α in cell supernatants were measured by ELISA in these three groups. *P < 0.05, **P < 0.01.

## Discussion

Recently, the cases of liver IR injury are increasing with the occurrence of diseases in liver [30]. Although crucial advances have been achieved in treatment strategies, the risk of IR injury still exists and threatens the life of patients. Hence, it is necessary to discover novel methods to improve the treatment results.

Accumulating studies have suggested that MALAT1 could function as a key effector in regulating the biological processes in various diseases. Specifically, MALAT1 targets miR-188-5p to affect cell proliferation and apoptosis in multiple myeloma [31]. MALAT1 knockdown is reported to protect against intracerebral hemorrhage via miR-146a [32,33]. Herein, we explored into the implication of MALAT1 during liver IR injury. First, we built the IR and H/R model and found that the MALAT1 level was the highest after 6-h reperfusion treatment. On this basis, we carried out loss of functional assays in vitro with H/R model and primary mouse hepatocytes extracted from IR model to investigate the effects of MALAT1 on IR injury. Data manifested that downregulated MALAT1 promoted cell viability and repressed apoptosis rate and inflammatory reaction in liver IR injury, suggesting the promoting role of MALAT1 in liver IR injury.

Existing report has unveiled that lncRNAs could function as a ceRNA in modulating the progression of diseases including IR injury [16]. Additionally, MALAT1 has been reported to target miR-144-3p and thus contribute to apoptosis in myocardial infarction [34] and affect cardiomyocyte apoptosis after hypoxia/reperfusion injury through modulation on miR-200a-3p/PDCD4 [35]. Additionally, MALAT1 enhances cell apoptosis and impedes cell proliferation in testicular IR injury via targeting miR-214/ TRPV4 [36]. Consistently, our study also confirmed that MALAT1 acted as a ceRNA to target miR-150-5p in liver IR injury. Moreover, we also detected the expression of miR-150-5p in H/R model and found that miR-150-5p level was lowered after 6-h treatment of reoxygenation. MiR-150-5p has been identified to exert inhibitory influences on nasopharyngeal carcinogenesis by suppressing PYCR1 [37]. In line with previous study, our research also identified that miR-150-5p inhibited the progression of liver IR injury through gain of function assays.

RETRACTED

Hinted by published reports revealing that lncRNA could take part in the ceRNA mechanism via sequestering miRNAs to regulate target genes [38], the downstream mRNA of MALAT1/miR-150-5p was also taken into consideration. Based on bioinformatics analysis and mechanism assay results, AZIN1 was sustained as the downstream of miR-150-5p and was negatively modulated by miR-150-5p. More importantly, we conducted rescue experiments and verified that AZIN1 upregulation could neutralize the impacts of MALAT1 silence on the progression of liver IR injury.

To summarize, the function and potential regulatory mechanism of MALAT1 implicated in both IR model and H/R model were verified. Although MALAT1 has been discovered as a gene affecting cerebral IR injury through ceRNA mechanism [39], it was the first to confirm that MALAT1 accelerated the proliferation, apoptosis, and inflammatory reactions in liver IR injury model by targeting miR-150-5p/AZIN1 axis. These findings together indicated that MALAT1 might be a potential therapeutic target for the treatment of liver IR injury.

## Conclusion

MALAT1 was upregulated in the IR model and H/R model. MALAT1 depletion caused enhanced viability and weakened apoptosis and inflammation of H/R-treated cells. Mechanism assays along with functional assays jointly proved that MALAT1 regulated miR-150-5p/AZIN1 to affect cell proliferation, apoptosis, and inflammatory reactions, thus exacerbating liver IR injury.

## Supplementary Material

Supplemental Material
